# Psorachromene Suppresses Oral Squamous Cell Carcinoma Progression by Inhibiting Long Non-coding RNA GAS5 Mediated Epithelial-Mesenchymal Transition

**DOI:** 10.3389/fonc.2019.01168

**Published:** 2019-11-05

**Authors:** Tong-Hong Wang, Yann-Lii Leu, Chin-Chuan Chen, Tzong-Ming Shieh, Jang-Hau Lian, Chi-Yuan Chen

**Affiliations:** ^1^Tissue Bank, Chang Gung Memorial Hospital, Tao-Yuan, Taiwan; ^2^Research Center for Chinese Herbal Medicine, Graduate Institute of Health Industry Technology and Research Center for Food and Cosmetic Safety, College of Human Ecology, Chang Gung University of Science and Technology, Tao-Yuan, Taiwan; ^3^Department of Hepato-Gastroenterology, Liver Research Center, Chang Gung Memorial Hospital, Tao-Yuan, Taiwan; ^4^Graduate Institute of Natural Products, Chang Gung University, Tao-Yuan, Taiwan; ^5^Chinese Herbal Medicine Research Team, Healthy Aging Research Center, Chang Gung University, Tao-Yuan, Taiwan; ^6^Center for Traditional Chinese Medicine, Chang Gung Memorial Hospital, Tao-Yuan, Taiwan; ^7^Department of Dental Hygiene, China Medical University, Taichung, Taiwan; ^8^Genomic Medicine Core Laboratory, Chang Gung Memorial Hospital, Tao-Yuan, Taiwan

**Keywords:** psorachromene, oral squamous cell carcinoma (OSCC), long non-coding RNA, growth arrest-specific transcript 5 (GAS5), epidermal growth factor receptor (EGFR)

## Abstract

The extract of the seeds of *Psoralea corylifolia* Linn. (*P. corylifolia*) have been shown to display anti-tumor activity. However, the prospects of the active compounds from this plant in the treatment of oral squamous cell carcinoma (OSCC) remains unclear. In the present study, the antitumor effects of psorachromene, a flavonoid extracted from the seeds of *P. corylifolia*, were investigated using cells and animal models of OSCC; the downstream regulatory mechanisms were also elucidated. The results showed that psorachromene significantly repressed cell proliferation, migration, and invasiveness and increased the toxic effects of chemotherapeutic agents against OSCC cells. The repressive effects of psorachromene were attributable to the inhibition of EGFR-Slug signaling, and the induction of G2/M arrest and apoptosis in the OSCC cells. Additionally, we found that psorachromene induced the expression of tumor suppressor long non-coding ribonucleic acid (RNA) growth arrest-specific transcript 5 (GAS5) and the activation of its downstream anticancer mechanisms. Animal experiments also showed noticeable inhibition of tumor growth, without significant physiological toxicity. The findings indicate that psorachromene displays anti-tumor activity in OSCC, and warrants further investigation as a potential agent for clinical application.

## Introduction

Oral cancer is the eleventh most common malignancy worldwide (1). In Taiwan, more than 4,700 people are diagnosed with oral cancer each year, and ~2,200 people die from it. Among all types of oral cancer, oral squamous cell carcinoma (OSCC) is the most common, with an incidence of ~90% (2). Smoking, drinking alcohol, and chewing tobacco or betel seeds are risk factors for OSCC (3–5). Currently, the mainstay treatment for OSCC is surgical resection, with adjuvant chemotherapy or radiotherapy (6, 7). In addition, epidermal growth factor receptor (EGFR) and cyclooxygenase-2 (COX-2) inhibitors are also used in the treatment of OSCC (8, 9). However, the benefits of these therapies remain sub-optimal, and their side effects have a considerable impact on patients' quality of life. Therefore, oral cancer research continues to focus on the development of effective new treatment methods with minimal side effects.

Cancer-causing gene mutations are one of the major causes of OSCC (10–12). Previous studies have shown that over 75% of OSCC shows epidermal growth factor receptor (EGFR; also known as ErbB1 or HER1) overexpression; EGFR expression has shown a significantly positive association with the degree of malignancy (13–15). Therefore, inhibiting the growth of cancer cells by EGFR signaling inhibition is one of the current treatment strategies for OSCC (16, 17). Various EGFR inhibitors including anti-EGFR monoclonal antibodies (cetuximab and panitumumab) and small-molecule EGFR tyrosine kinase inhibitors (gefitinib, afatinib, and erlotinib) have been developed, and have demonstrated efficacy in OSCC (16, 18–20). However, only the monoclonal antibody cetuximab is currently approved for the treatment of OSCC; it has demonstrated significant inhibition of the progress of OSCC, with extension of survival (21, 22). Unfortunately, for reasons that are not fully clear, only ~50% of patients respond to cetuximab (23, 24).

Traditional Chinese medicine (TCM) has long been used for the treatment of diseases in Asian countries (25, 26). Unlike Western medicine, TCM provides effective treatment options with relatively milder adverse effects (27–29). However, differences in the quality of TCM therapeutics and the levels of active ingredients usually result in variable therapeutic effects (30). In order to achieve more stable therapeutic effects, the active ingredients of many traditional Chinese medicinal materials have been purified and identified (31–33). The identified compounds can be used at lower doses with more specific therapeutic efficacy. Currently, many compounds extracted from TCM therapeutics, e.g., artemisinin, curcumin, resveratrol, and paclitaxel, which are used in the treatment of cancer have shown good efficacy (34–38). Among them, paclitaxel, camptothecin, and vinblastine, have also been approved for the treatment of various cancers, including lung cancer, liver cancer, and oral cancer (39).

*Psoralea corylifolia* L. is a TCM herb that is commonly used in Asian countries for the treatment of bacterial infections, inflammation, and cancer (40–44). *P. corylifolia* L. contains flavonoids such as bavachin, isobavachalcone, and neobavaisoflavone; polyphenols such as psoralidin, psoralen, and isopsoralen; and benzene ring compounds such as backuchiol; in addition, the herb has been found to have biological activity and various therapeutic effects (42). Psorachromene is an isoflavone component isolated from the fruit kernels of *P. corylifolia* L. (45). A few studies have investigated the mechanism of action of psorachromene. Recent reports indicate that psorachromene has anti-inflammatory effects that may inhibit inflammatory reactions caused by inducible NO synthase (iNOS) and cyclo-oxygenase (COX) expression induced by bacterial infection (46). However, there have been no studies on its anticancer effects. In this study, we investigated the anticancer activity of psorachromene in oral cancer, and studied its downstream regulatory mechanisms.

## Materials and Methods

### Cell Lines and Culture Media

SAS is a human tongue squamous cell carcinoma cell line from the Japanese Collection of Research Bioresources (Tokyo, Japan) (47). OECM1 is a Taiwanese human gingival squamous carcinoma cell line; its derivation has been described in a previous study (47). Both cell lines were cultured in Dulbecco's modified Eagle's medium (DMEM) containing 10% fetal bovine serum (FBS), 1.2 g/L sodium bicarbonate, 0.5 mM sodium pyruvate, and 2.5 mM L-glutamine. The culture media, FBS, and chemical compounds were purchased from Life Technologies (Grand Island, NY, USA). The cells were cultured at 37°C in a humidified 5% CO_2_ incubator.

### Reagents and Antibodies

The crude materials of the *P. corylifolia* seed were purchased from Chuang Song Zong Pharmaceutical Co., Ltd (Kaohsiung, Taiwan). The dried seeds of *P. corylifolia* were infused in ethanol and were filtered to obtain the crude extract. The crude extract was partitioned in n-hexane/water (1:1). The n-hexane soluble extract was then fractionated by column chromatography on silica gel, eluting with n-hexane: ethylacetate to isolate psorachromene. The purity of psorachromene was determined by nuclear magnetic resonance analysis. Antibodies against vimentin, E-cadherin, slug, cleaved-PARP (cl-PARP, Asp214), and caspase 9 were obtained from Cell Signaling (Temecula, CA, USA). Antibodies against EGFR and β-actin were purchased from Santa Cruz Biotechnology (Santa Cruz, CA, USA). Prestained protein marker and TOOLSmart RNA extractor were purchased from BIOTOOLS (New Taipei City, Taiwan). The cisplatin and doxorubicin were purchased from Sigma-Aldrich (St. Louis, MO, USA), and the reagents for gel electrophoresis were purchased from Bio-Rad (Berkeley, CA, USA).

### Cell Viability Assays

Cell viability was determined using the sulforhodamine B (SRB) assay by staining with trypan blue, as described previously (48, 49).

### Terminal Deoxynucleotidyl Transferase dUTP Nick End Labeling (TUNEL) Assay

The apoptotic status of the treated cells was determined using a DeadEnd^TM^ Fluorometric TUNEL Assay Kit (Promega, Madison, WI) according to the manufacturers' protocol. In summary, the SAS cells were treated with psorachromene (50 μM) for 24 h and were then subjected to a terminal deoxynucleotidyl transferase dUTP nick end labeling (TUNEL) assay. The apoptotic cells (DAPI and TUNEL double stained cells) were enumerated using a fluorescence microscope (magnification, × 100). Cells in five different microscopic fields/dish were analyzed for each experiment.

### Western Blotting

Cells were washed twice with phosphate-buffered saline (PBS), lysed in 200 μL of RIPA lysis buffer (Biotools Co. Ltd., Taiwan) containing protease inhibitors, and incubated on ice for 10 min. The samples were then centrifuged at 12,000 rpm for 30 min at 4°C, and the protein-containing supernatants were collected. The protein concentrations were determined using the Bio-Rad protein assay, and western blotting was performed as described previously (49).

### Phenotypic Analysis for Clonogenic, Migration, and Invasion Ability

The clonogenic, migration, and invasion assays were performed as described previously (47).

### Cell-Cycle Analysis

Cells were trypsinized, washed twice, and incubated in PBS containing 0.12% Triton X-100, 0.12 mmol/L EDTA, and 100 mg/mL ribonuclease A. Propidium iodide (50 μg/mL) was then added to each sample, and they were kept at 4°C for 20 min. Cell cycle distribution was then analyzed using flow cytometry (Beckman Coulter Epics Elite, Beckman, Inc.).

### Whole-Transcriptome Sequencing

RNA extraction and whole-transcriptome sequencing was performed as described in a previous study (25).

### Detection of lncRNA GAS5

RNA from the cells were isolated using a RNeasy mini kit (QIAGEN, Gaithersburg, MD, USA), according to the manufacturer's instructions. Two micrograms of RNA sample were subjected to reverse transcription (RT) using the reverse transcription kit (Applied Biosystems, Foster City, CA, USA). The expression of lncRNA GAS5 was detected by quantitative polymerase chain reaction (PCR) using the TaqMan gene expression assay (Applied Biosystems, Foster City, CA, USA), as described previously (50). Glyceraldehyde 3-phosphate dehydrogenase (GAPDH) was used as an internal control.

### RNA Interference (RNAi)

Human lncRNA GAS5 were downregulated using a mixture of four small interfering RNAs (siRNAs) (ON-TARGETplus SMARTpool; Dharmacon, Lafayette, CO) as previously described (50). In summary, the four siRNAs targeting lncRNA GAS5 (GenBank accession no. NR_002578.2) covered the following: nucleotides 385-403 from the start codon (lncRNA GAS5-1: AGGCAGACCUGUUAUCCUA), nucleotides 248-266 (lncRNA GAS5-2: UGGAUGACUUGCUUGGGUA), nucleotides 567-585 (lncRNA GAS5-3: GAUGGAGUCUCAUGGCACA), and nucleotides 301-319 (lncRNA GAS5-4: AGGUAUGGAGAGUCGGCUU). Transfection was performed using the Dharmafect 1 transfection reagent (Dharmacon) according to the manufacturer's instructions.

### *In vivo* Tumor Xenograft Study

The *in vivo* antitumor activity of psorachromene against SAS cells was studied using 6-week-old nude BALB/c nu/nu male mice. SAS cells (5 × 10^5^) were subcutaneously implanted in the right flank of the mice on day 0. The mice were then randomized on day 7 into vehicle control and treatment groups of six animals each. Psorachromene and cisplatin were administered intraperitoneally thrice weekly, with 100 μL of psorachromene (25 mg/kg of body weight), cisplatin (2 mg/kg), or an equal volume of dimethyl sulfoxide (DMSO), which served as a control. The tumor volume was evaluated every 2 days using calipers, based on the following formula: tumor volume = length × width^2^/2. Their body weights and food consumption were also determined to evaluate apparent signs of toxicity. The tumor-bearing mice were weighed and sacrificed on day 22 for assaying the tumor biology. All animal experiments were performed in accordance with the guidelines for the Animal Care Ethics Commission of the Chang Gung Memorial Hospital, under an approved animal protocol (IACUC approval no. 2018031301).

### Immunohistochemistry

The tumors were fixed in formalin and embedded in paraffin. Consecutive 2-μm-thick sections were obtained from the paraffin-embedded tissue blocks, and were floated onto glass slides. The slide-mounted tissue sections were subjected to immunohistochemical staining as described previously (51).

### Statistics

All data have been presented as means ± standard deviations (SD). The Student's *t*-test was employed for comparison, and all analyses were performed using the Statistical Package for the Social Sciences version 12.0 (SPSS, Inc.). Differences between the variables were considered significant for *p*-values of > 0.05.

## Results

### Psorachromene Inhibited the Growth of OSCC Cells and Promoted Their Apoptosis

Psorachromene is a flavonoid extracted from the seeds of *P. corylifolia* L. (Figure 1A). In this study, we treated OSCC cells and human fibroblast cell lines with different concentrations of psorachromene and analyzed the cell proliferation status using Sulforhodamine B (SRB) assay to determine whether psorachromene has inhibitory activity on OSCC. The results showed that psorachromene could significantly inhibit the growth of SAS and OECM1 cells starting from concentrations of 25 μM; the inhibitory effect became more significant with increasing psorachromene concentrations (Figure 1B). Similar results were obtained on the trypan blue staining assay. Psorachromene significantly inhibited the growth of SAS and OECM1 cells in a dose dependent manner. However, no inhibitory effect was observed on the growth of human fibroblast cell line HFB (Figure 1C). This indicated that psorachromene selectively inhibits the growth in OSCC cells without significant toxicity to normal cells. We also evaluated the impact of psorachromene on the colony forming ability of OSCC. The results showed significant inhibitory activity in a dose-dependent manner. At a concentration of 50 μM, psorachromene inhibited the colony forming ability of OSCC cells by more than 90% (Figures 1D,E), confirming its inhibitory activity on the growth of OSCC cells.

**Figure 1:** Inhibition of the proliferation of OSCC cells by psorachromene. **(A)** Chemical structure of psorachromene. SAS and OECM1 cells were treated with different concentrations of psorachromene or vehicle (DMSO), and the cell proliferation status was analyzed using the SRB assay **(B)**, trypan blue staining assay **(C)**, and colony formation assay **(D,E)**. The results are the mean of three independent experiments. Significant differences vs. the control groups, ^*^p < 0.05, ^***^p < 0.001.

To determine the mechanism of inhibition of OSCC, we further compared the cell cycle progression between cells treated and not treated with psorachromene. Those treated with psorachromene were found to have been arrested in the G2 phase, their numbers in the sub-G1 phase were significantly higher compared to the control group (Figures 2A,B). These findings suggested that psorachromene inhibits cell cycle progression and promotes cell apoptosis. The results of the TUNEL assay also demonstrated that the number of apoptotic cells in the psorachromene treatment group were significantly higher compared with the control group (Figures 2C,D). Furthermore, the results of western blotting analysis confirmed the activation of caspase-9 and the cleavage of poly (ADP-ribose) polymerases (PARPs) by psorachromene, indicating that it promotes cell apoptosis by activating apoptosis-related proteins (Figure 2E).

**Figure 2:** Inhibition of cell cycle progression and promotion of apoptosis in OSCC cells by psorachromene. **(A,B)** Effect of psorachromene on cell cycle progression in SAS and OECM1 cells. The cells were treated with vehicles or different concentrations of psorachromene for 24 h. Cell cycle distribution was analyzed by flow cytometry. **(C)** SAS cells were treated with or without psorachromene, and cell apoptosis was determined using a terminal deoxynucleotidyl transferase dUTP nick end labeling (TUNEL) assay. Green punctate staining (white arrows) represents TUNEL-positive cells. Apoptotic cells were identified as DAPI and TUNEL double-stained cells. Magnification: 100×. Quantitative results seen in **(D)**. **(E)** Western blot analysis showing the effect on caspase 9 and PARP activity in OSCC cells after 48 h of psorachromene treatment. ^*^p < 0.05, ^**^p < 0.01, ^***^p < 0.001.

### Psorachromene Inhibits the Migration and Invasiveness of OSCC

Invasion and metastasis are the major contributors to the refractory nature of cancer. We conducted a wound-healing assay to evaluate whether psorachromene may affect cell migration; this was performed to further evaluate the potential of psorachromene in inhibiting metastasis and invasiveness in OSCC cells. The results showed that at a concentration of 25 μM, psorachromene significantly inhibited cell migration ability, and the inhibitory effects increased with the concentration of psorachromene. At a concentration of 75 μM, psorachromene inhibited the migration ability of SAS and OECM cells by 51.3 and 19.1%, respectively (Figures 3A,B). Furthermore, the invasion assay demonstrated that psorachromene may inhibit cell invasion by up to 83.7% at a concentration of 75 μM (Figures 3C,D).

**Figure 3:** Inhibition of cell metastasis ability in OSCC by psorachromene by inhibition of the progression of epithelial-mesenchymal transition. **(A)** The effect of psorachromene on the wound-healing ability of SAS and OECM1 cells. Quantitative results are seen in **(B)**. **(C,D)** The effect of psorachromene on the invasiveness of SAS and OECM1 cells. **(E)** Western blotting was used to examine the levels of EMT regulatory proteins in OSCC cells treated with psorachromene for 48 h. The quantified results are shown in (**F**). ^*^p < 0.05, ^**^p < 0.01, ^***^p < 0.001.

### Psorachromene Inhibits Epithelial-Mesenchymal Transition (EMT)

Epithelial-mesenchymal transition (EMT) is an important process in cancer cell metastasis, that weakens intercellular adhesions and facilitates metastasis. To determine whether psorachromene regulates EMT when inhibiting OSCC migration and invasion abilities, we performed western blotting to analyze the effects of psorachromene on EMT associated proteins. The results indicated that the expression of EMT-promoting proteins such as vimentin and slug was significantly lower in psorachromene-treated cells compared with the control group. However, the expression of E-cadherin did not change significantly (Figures 3E,F), suggesting that psorachromene may inhibit OSCC migration and invasion by inhibiting EMT.

Slug is a downstream gene regulated by the EGFR signaling pathway. We also evaluated whether psorachromene affects EGFR expression, and found its expression in psorachromene-treated cells to be significantly lower compared to the control group (Figures 3E,F). The results indicated that psorachromene may inhibit the expression of slug, and the progression of EMT by downregulating EGFR expression.

### Psorachromene May Enhance the Therapeutic Effects of Cisplatin and Doxorubicin on OSCC

Cisplatin and doxorubicin are the commonly used chemotherapeutic drugs in the treatment of OSCC (52–54). In order to determine whether combining psorachromene with these drugs may improve their therapeutic effects on OSCC, we administered psorachromene, cisplatin, and doxorubicin alone, or in combination to the OSCC cells; we also evaluated its inhibitory effects on the growth of these cells. Cisplatin and doxorubicin alone had an inhibitory effect on OSCC; however, combination with psorachromene significantly enhanced the inhibition of OSCC. Compared to cisplatin or doxorubicin alone, the combination with psorachromene enhanced the toxicity on OSCC cells by up to 3.3-fold (Figures 4A,B). The combination index also demonstrated the additive effect of psorachromene in combination with cisplatin and doxorubicin (Table 1).

**Figure 4:** Psorachromene combined with cisplatin and doxorubicin has additive effect. The effects of psorachromene combined with cisplatin and doxorubicin on proliferation of SAS **(A)** and OECM1 **(B)** cells. ^*^p < 0.05, ^**^p < 0.01, ^***^p < 0.001. All experiments were performed in triplicate.

**Table 1:** The combination index.

	**PC (μM)**	**DOX (μM)**	**CI**
SAS	25	0.05	0.68011
	25	0.1	0.50582
	50	0.05	1.04119
	50	0.1	0.84218
OECM1	25	0.05	0.79836
	25	0.1	1.18195
	50	0.05	1.51916
	50	0.1	1.84227
	**PC (μM)**	**CIS (μM)**	**CI**
SAS	25	25	0.99174
	25	50	0.63005
	50	25	0.96329
	50	50	0.75840
OECM1	25	5	1.93719
	25	25	0.84726
	50	5	0.84689
	50	25	0.76593

### Psorachromene Inhibits Tumor Growth in Mice

The anticancer effects of psorachromene *in vivo* were verified using a mouse xenograft model; the effects of psorachromene on tumor growth in mice were similar to those of the cell experiments. The tumor growth rate was significantly reduced in mice treated with psorachromene. After 2 weeks of administering the drug, the tumor volume in the psorachromene-treated group was reduced by ~75.5% compared with the control group (Figures 5A,B), and the tumor inhibitory effect was equivalent to that of the cisplatin-treated group (84.6%). In addition, there were no significant differences in body weight between the psorachromene-treated and control groups (Figure 5C), indicating that psorachromene may not have significant physiological toxicity.

**Figure 5:** Psorachromene inhibits tumor growth in mice. **(A)** A total of 5 × 10^6^ SAS cells were inoculated into nude mice (*n* = 6). Representative images show the tumor xenografts at 3 weeks after implantation. Psorachromene significantly reduced tumor growth. **(B)** Tumor volumes were calculated every 3 days after injection. The volume of each tumor was calculated as follows: length × width^2^ × 0.5. Bars indicate S.D. ^***^p < 0.001. **(C)** Body weights were calculated every 3 days after injection. **(D)** Immunohistochemical staining represents the effect of psorachromene on the expression of EGFR and EMT associated proteins in mice xenograft tumors. Magnification: 400×.

In addition, we analyzed the expression of EGFR and EMT-related proteins including slug, vimentin, and E-cadherin in murine tumor tissues using immunohistochemical staining, and found that psorachromene may significantly inhibit the expression of EGFR and EMT-promoting proteins (Figure 5D). The results of this experiment were identical to those of cellular experiments, suggesting that psorachromene may inhibit EMT.

### Psorachromene May Inhibit the Activation of Signaling Pathways Associated With Cell Growth and Extracellular Structure Organization

To understand its anticancer mechanisms of action, we treated SAS and OECM1 cell lines with psorachromene, and performed whole-transcriptome sequencing to identify the genes and signaling pathways that may be regulated by psorachromene. Heatmap analysis showed that after psorachromene treatment, gene expression was significantly altered compared with the control group (Figure 6A). We further performed ingenuity pathway analysis, and found that psorachromene mainly regulates the LKB1 and ErbB/EGFR signaling pathways (Figure 6B), affects the energy metabolism of cells, and the composition and generation of the extracellular matrix, thereby inhibiting their growth and metastasis.

**Figure 6:** Psorachromene-induced regulation of gene expression related to cell growth and extracellular structure organization. **(A)** Heatmap comparing significantly different expression of genes in SAS and OECM1 cells treated with or without psorachromene. The bar charts represent the enriched biological pathways **(B)** associated with the differentially expressed genes after psorachromene treatment. **(C)** The whole-transcriptome sequencing data shows that 12 lncRNAs manifested higher than a 2-fold change in expression after psorachromene treatment in both cell lines. **(D)** SAS and OECM1 cells were treated with psorachromene for 48 h, and GAS5 expression was analyzed using quantitative real-time RT-PCR. ^*^p < 0.05, ^***^p < 0.001.

### Psorachromene Exerts Anticancer Effects by Inducing the Expression of Long Non-coding RNA GAS5

Previous studies have confirmed that long non-coding RNAs (lncRNAs) play an important role in cell physiological regulation, and drug responses. To understand the role of lncRNAs in the anti-OSCC mechanisms of action of psorachromene, we analyzed the previously-mentioned transcriptome sequencing data, and found that 12 lncRNAs demonstrated a higher than 2-fold change in expression after psorachromene treatment, compared to the control group (Figure 6C). Among these lncRNAs, growth arrest-specific transcript 5 (GAS5) has recently been discovered to suppress cancer. It has been shown to inhibit the growth and metastasis of OSCC by regulating the miR-21/PTEN axis. To confirm the regulatory relation between psorachromene and GAS5, we performed real-time reverse transcriptase-PCR to determine the expression of GAS5 in OSCC cells. The results indicated that the expression of GAS5 in SAS and OECM1 cells treated with psorachromene was significantly higher than that of the control group (Figure 6D); this indicates that psorachromene may inhibit the growth and metastasis of OSCC by inducing GAS5 mediated anticancer mechanisms.

We performed a rescue assay to further verify the mentioned conditions. The results showed that psorachromene significantly inhibited the growth and migration of OSCC cells. After silencing GAS5 expression, we found that the inhibitory effects of psorachromene on OSCC cells were attenuated (Figures 7A–D); this indicated that the anti-OSCC action of psorachromene is partly achieved by regulating the lncRNA-GAS5 anticancer pathway.

**Figure 7:** The anticancer effect of psorachromene is exerted by inducing expression of lncRNA-GAS5. **(A)** Real-time PCR analysis shows the effect of siRNA treatments on the expression of GAS5 in OECM1 cells. GAPDH served as an internal control. **(B,C)** The inhibitory effects of psorachromene on cell proliferation and migration were significantly reversed by treatment with GAS5 siRNA (50 nM) in the OECM1 cells. The quantitative cell migration result was shown in **(D)**. ^*^p < 0.05, ^**^p < 0.01, ^***^p < 0.001.

## Discussion

Psorachromene is a flavonoid component of *P. corylifolia* L., accounting for 0.0016% of the total extract from the seeds of *P. corylifolia* L (55). Current understanding on the biological functions of psorachromene is limited. Only a few studies have reported on its anti-inflammatory activity, which may inhibit inducible nitric oxide synthase (iNOS) and COX expression induced by lipopolysaccharide (LPS), thereby inhibiting inflammatory reaction (46). However, no studies have evaluated its anticancer effects. In this study, we investigated the inhibitory activity of psorachromene on OSCC, and found that it significantly inhibited the growth, migration, and invasiveness of OSCC cells, and suppressed EMT by inducing the expression of lncRNA-GAS5. The results of our animal experiments also showed that it may significantly inhibit the growth of tumor cells and the expression of EMT-associated proteins. To the best our knowledge, this is the first study to demonstrate that psorachromene regulates lncRNAs to exert its antitumor effects.

Previous studies have shown that ~80% of OSCC over-express EGFR; this leads to uncontrolled cell growth and enhances the metastatic ability of the cells (13, 56). It also enhances the resistance of OSCC to chemotherapeutic drugs including, cisplatin, 5-fluorouracil (5FU), and doxorubicin (57–59). Previous studies have also confirmed that the use of the EGFR inhibitor gefitinib in combination with cisplatin enhanced the therapeutic effects of the latter on OSCC (20). This study demonstrated similar results. In addition to the inhibition of EGFR expression, psorachromene has synergistic activity with cisplatin and doxorubicin in the treatment of OSCC, with no significant physiological toxicities. Therefore, psorachromene has considerable potential for use as a therapeutic adjuvant in the treatment of OSCC.

To identify the genes and anticancer signaling pathways that may be regulated by psorachromene, we performed whole-transcriptome sequencing that examined the gene expression profiling of psorachromene in treated and untreated cells. The results showed that psorachromene mainly regulates the expression of genes associated with cell growth, extracellular matrix composition, and inflammation, among others, thereby inhibiting the growth and metastasis of OSCC cells; this was consistent with the results observed on cell functional assay. The inhibitory effect of psorachromene on the Erb-1 pathway indicates that it has considerable potential in the treatment of cancers that overexpress EGFR (including cancers of the breast and liver); it may also synergize with other anticancer drugs to enhance their therapeutic efficacy.

This study revealed that psorachromene induces lncRNA-GAS5 expression, which is a known anticancer lncRNA, and participates in the regulation of many important physiological processes, including cell growth, apoptosis, cell cycle progression, and EMT (60, 61). The low expression of GAS5 is closely related to the poor prognosis and chemoresistance of many cancers (62–65). Overexpression of GAS5 could enhance the inhibitory effect of Gefitinib on EGFR phosphorylation and its downstream signaling activation, while enhancing the sensitivity of lung cancer cells to EGFR-TKI (66). In addition, the chemotherapeutic drug, Lapatinib, can also enhance the response of breast cancer cells to trastuzumab by inducing GAS5 expression (67). Some studies have also suggested that GAS5 is significantly downregulated in OSCC cells, and that GAS5 expression may inhibit the growth and metastasis of OSCC by regulating the miR-21/PTEN axis (68). In this study, we found that psorachromene may induce GAS5 expression. It is speculated that the inhibitory effects of psorachromene on OSCC are partly attributable to GAS5-mediated anticancer mechanisms. Moreover, this result also shows the potential of psorachromene as a therapeutic adjuvant that enhances the sensitivity of cancer cells to chemotherapeutic drugs by inducing the expression of GAS5.

Previous studies have demonstrated that long non-coding RNAs are involved in the regulation of a wide range of gene expression or protein stability. However, recent studies have shown that GAS5 does not regulate EGFR expression (66). We speculate that psorachromene regulates GAS5 and EGFR expression through two independent mechanisms; however, the detailed regulatory mechanism is yet to be delineated. In addition, the results of whole-transcriptome sequencing analysis showed that numerous lncRNAs are also regulated by psorachromene; the role of these lncRNAs in the anticancer mechanisms of psorachromene warrant further research.

In cell cycle analysis related to psorachromene treatment, the distribution of cell cycle between SAS and OECM1 cells is quite different. The inhibitory effect of psorachromene on SAS cells is better than that of OECM1. We speculated that the anti-OSCC effect of psorachromene may be induced by specific receptors. The genetic background difference between cells leads to the differences in receptor expression, which affect the anti-OSCC effect of psorachromene. However, the receptor that is targeted by psorachromene to achieve its anticancer mechanism and its detailed downstream regulation mechanism still need to be clarified to improve the clinical applicability of psorachromene.

The concentrations of psorachromene in *P. corylifolia* L. are not high; in addition, it has a simple structure. Therefore, psorachromene is mainly synthesized chemically for commercial formulations. Structural modifications may be introduced in the future to increase its anticancer activity and intracellular availability. In this study, we demonstrated the potential anticancer activity of psorachromene using cell and animal experiments; we also found that it affects certain relevant regulatory pathways. The small-molecule compounds that are commonly used in clinical practice only block specific carcinogenic pathways; in contrast, psorachromene has a wide range of targets. In addition, the animal experiments did not demonstrate significant differences in physiological toxicity compared to these molecules. In view of these findings, psorachromene holds promise as a new therapeutic agent for OSCC. Further studies with larger sample sizes are needed to validate our findings.

## Data Availability Statement

The data for this manuscript has been uploaded to: https://www.ncbi.nlm.nih.gov/bioproject/PRJNA562818.

## Ethics Statement

The animal study was reviewed and approved by Animal Care Ethics Commission of the Chang Gung Memorial Hospital (IACUC approval no. 2018031301).

## Author Contributions

C-YC, T-HW, and Y-LL contributed to the conception and design of the study. C-YC, T-HW, Y-LL, C-CC, T-MS, and J-HL performed the experiments and statistical analyses. T-HW and C-YC prepared the first draft of the manuscript. All authors contributed to manuscript revision and have read and approved the submitted version.

### Conflict of Interest

The authors declare that the research was conducted in the absence of any commercial or financial relationships that could be construed as a potential conflict of interest.
